# *In vitro* maturation of *Mus musculus* mice oocytes after hyperosmotic shock induced by vitrification solutions

**DOI:** 10.5935/1518-0557.20200084

**Published:** 2021

**Authors:** Erica Koaski, Cláudia Schneider Colle, Rafael Alonso Salvador, Vera Lucia Lângaro Amaral, Alfred Paul Senn, David Til

**Affiliations:** 1 Universidade do Vale do Itajaí (UNIVALI), Laboratory of Reproductive Biology, Itajaí/SC, Brasil; 2 Fertas Brasil, Balneário Camboriú/SC, Brasil

**Keywords:** Oocyte maturation, oocytes, hyperosmotic shock, meiosis resumption, mice

## Abstract

**Objective:**

To evaluate *in vitro* oocyte maturation rates in embryonic culture medium after induction by hyperosmotic shock caused by exposure to vitrification solutions.

**Methods:**

Bilateral oophorectomy was performed on 20 prepubescent female mice (Swiss). Immature (Prophase I) oocytes (N = 400) were obtained by ovarian dissection, divided into 4 groups, and transferred to culture dishes containing fertilization medium (Sydney IVF Fertilization Medium, Cook^®^ Medical). The control group (CG) did not receive treatment, the test groups (G1, G2, G3) were treated with vitrification solution - 2 (VI-2: 14 M sucrose + ethylene glycol and dimethyl sulfoxide) for 30 seconds and subsequently: G1: 30 seconds in devitrification solution - 2 (DV-2: 0.5M sucrose); G2: 60 seconds DV-2; G3: 60 seconds DV-1(1M sucrose) and 180 seconds DV-2. All groups were cultivated for 24 hours in an incubator at 37ºC and 5% CO2 (Thermo model 3110). After this period, we checked their maturation status.

**Results:**

Oocytes exposed to VI-2, DV-1 and DV-2 (G3) showed the highest rate of competence in resuming meiosis and reaching the MII stage; however, there was no statistically significant difference (G3 = 50.5% - 49/97; CG = 27.8% - 10/30).

**Conclusions:**

Oocyte exposure to vitrification solutions, in order to cause osmotic shock, did not interfere with the resumption of meiosis in mice oocytes.

## INTRODUCTION

Despite the significant progress of cancer treatments, the quality of patients’ survival may be reduced by the occurrence of early gonad functional failure, leading to infertility (Matos et al., 2012; Mandinka et al., 2014). Consequently, the concern with the quality of life after cancer treatment boosted the exploration of means to preserve fertility, especially among younger patients who might be adversely affected before having given birth to an offspring or reached reproductive age (Carvalho, 2015). Using assisted reproduction techniques, it is now possible to induce viable pregnancies in infertile patients (Félis & Almeida, 2016), but also to preserve fertility in oncological patients undergoing chemotherapy or radiotherapy treatments (Tomás *et al*., 2016).

In adult patients, fertility preservation may be achieved through cryopreservation of embryos, oocytes or ovarian tissue (Carvalho *et al*., 2017; Matos *et al*., 2011). In prepubescent girls or in adult females who cannot receive hormonal stimulation due to the development of hormone-dependent tumors, leukemia or advanced diseases (Tomás *et al.*, 2016), cryopreservation of ovarian tissue is the only option (Mendonça *et al*., 2014). This technique still present some risks such as tissue ischemia or the development of tumors after reimplantation (Rosa e Silva, 2006). In this context, the collection of immature oocytes (in prophase I) for *in vitro* maturation (IVM) becomes an option that eliminates most of the disadvantages when compared to the existing approaches, since it is not necessary to suspend chemotherapy treatment, it does not require a partner or semen donor, and the patient does not need to have gone through puberty (Rosa e Silva, 2006).

The purpose of IVM is to simulate the *in vivo* process, giving the oocytes the necessary growth factors and hormones in order to allow them to restart meiosis and reach the metaphase II stage (Watson, 2007; Xu *et al*., 2009). Around birth, female germ cells are arrested in prophase of the first meiotic division. The oocytes remain blocked, until they are stimulated to mature and grow, an event that starts at puberty (Frantz *et al*., 2006). *In vivo*, the resumption of meiosis occurs through the action of the luteinizing hormone (LH), whereas, *in vitro*, it is only necessary to remove the oocyte from the follicle, in order to initiate nuclear maturation (Dekel *et al*., 1981).

Animal models provide useful information on the way substances may inhibit oocyte maturation, such as cyclic adenosine monophosphate (cAMP), or positively affect cell cycle, like proteins, growth factors, GnRH, purines, steroids, gonadotropins (Dieleman *et al*., 2002). The Ca2+ chelators block germinal vesical break down in mammalian oocytes at least up to the first metaphase. Furthermore, in absence of intracellular Ca2+ elevation, spontaneous meiosis resumption in vitro does not occur (Molina *et al*., 2016). Moreover, it has been demonstrated for Jones *et al*. (1995) that the injection of Ca2+ in mice oocytes induces parthenogenetic activation and subsequent normal embryo development. It is currently known that cryoprotectants such as dimethyl sulphoxide (DMSO) and ethylene glycol (EG) improve calcium transport in several cell lines (Castro *et al*., 2011). DMSO is known also to act on the release of calcium from intracellular storages and EG on its influx (Larman *et al*., 2006), which suggests that these compounds might be beneficial for oocyte maturation *in vitro*. IVM protocols have changed little over the past decades, and there is a growing interest in the clinical application of this technique in assisted reproduction (Coticchio *et al*., 2012).

The aim of this study is to evaluate the effect of hyperosmotic shock, caused by short exposure to cryopreservation solutions of immature oocytes from prepubescent mice, on the rates of oocyte maturation *in vitro*.

## MATERIAL AND METHODS

Animal experimentations were performed while respecting the norms recommended by the Brazilian Society of Science with Laboratory Animals (SBCAL) and the National Council of Control of Animal Experimentation (CONCEA). The experimental protocol was approved by the Ethics Committee for the Use of Animals of the Universidade do Vale do Itajaí (CEUA/UNIVALI) under protocol number 069/17.

Twenty prepuberal female mice (Mus musculus) of the Swiss lineage, 4 to 6 weeks old, were obtained from the Central Vivarium of the Universidade do Vale do Itajaí. The animals were kept in groups of 5 in polypropylene boxes, containing wood shavings and environmental enrichments (paper towels, boxes, rolls, and paper reels) in order to promote their well-being. Room temperature was maintained at 22±2ºC, under a photoperiod of 12 hours (light/dark). Water and food were provided *ad libitum*.

To perform bilateral oophorectomy, the female mice were slaughtered in a CO2/O2 chamber (Walls et al., 2015) using a proportion of 30% of CO2 and 70% of O2, aiming to reduce suffering, as recommended by the Ethics Committee for the Use of Animals. The ovaries were collected in a Petri dish containing buffered medium (GV-Hepes, Ingámed^®^, Maringá/PR, Brazil) and sectioned radially with a microneedle (0.45 x 13 mm, BD Medical, Brazil). The released immature oocytes were then retrieved and selected using a stereomicroscope (40x, Olympus SZ, Japan) based on their spherical shape, homogeneous cytoplasm, and lack of inclusions. The oocytes were immediately transferred to culture dishes (35 mm diameter, Ingámed^®^, Maringá/PR, Brazil) containing microdroplets of pre-equilibrated (5% CO2, 37 ºC) culture medium (Sydney IVF Fertilization Medium, CookMedical^®^, Australia).

We then divided the oocytes into 4 groups (CG n=108, G1 n=98, G2 n=97, G3 n=97). The experimental groups were exposed to vitrification/devitrification solutions for different time durations (Figure 1). Vitrification (VI-2, containing 0.5M sucrose, 15% EG, and 15% DMSO)and devitrification (DV-1, containing 1M sucrose; DV-2, containing 0.5M sucrose) solutions were obtained from Ingámed^®^. The control group (CG) was placed directly in culture without exposure to cryoprotectants. The G1 group was exposed to VI-2 (30 sec) followed by DV-2 (30 sec). The G2 group was exposed to VI-2 (30 sec) and to DV-2 (60 sec). The G3 group was exposed to VI-2 (30 sec), followed by DV-1 (60 sec) and DV-2 (180 sec). All groups were then cultivated for 24h at 37ºC under 5% CO2 (Thermo model 3110, Thermo Fisher Scientific, United States). After this period, we checked the oocyte maturation status.

**Figure 1:** Scheme of the methodology used in the study. In vitro oocyte maturation was performed in microdroplets of 30µL of Sydney IVF Fertilization Medium at 37ºC, 5% CO_2_ and high humidity. VI-2: vitrification solution, DV-1, and DV-2: devitrification solutions containing 1M and 0.5M sucrose respectively (Ingámed^®^) were used to induce a temporary hyperosmotic shock. N: number of immature oocytes in each group.

The characteristics indicative of nuclear maturation were scored as follows: 1) prophase I, presence of germinal vesicle (VG), 2) first meiotic metaphase (MI), absence of the nuclear membrane, 3) second meiotic metaphase (MII), presence of the first polar body in the perivitelline space (Setti *et al*., 2011). The following morphological aspects were also recorded: ooplasm sphericity, cytoplasm homogeneity, and the presence of inclusions. Oocyte morphology was good when the oocyte had a spherical shape and a homogeneous cytoplasm without inclusions (Setti *et al*., 2011). Calculated survival rates were based on oocytes with good morphology, observed only under the microscope, without any type of staining, throughout the IVM process. We calculated the rates of oocyte maturation reaching the stages of MI and MII after 24h.

We assessed the results by analyzing the ANOVA variance with the Tukey’s post-test (GraphPad software for Windows, San Diego, USA), and the differences were considered significant when *p*<0.05.

## RESULTS

Table 1 depicts the rates of oocytes maturation to MII stages. In the control group, 27.8% of immature oocytes reached the MII stage after 24h of IVM. In the G1, G2 and G3 groups the maturation rates were significantly higher (*p*<0.05) compared to the control group and reached 49.0%, 44.3%, and 50.5%, respectively. Among the treated groups, G3 produced higher maturation rates than G1 and G2, but with no statistically significant difference between the groups.

**Table 1:** Oocyte maturation rates of the control group and experimental groups (G1, G2, and G3) after hyperosmotic shock, induced by exposure to vitrification solutions. MII: number (n) of oocytes reaching the MII stages after 24h IVM. MI: number of oocytes (n) that reached the MI stage at some time point during IVM, this value includes both those, which remained at the MI stage after 24h, and those, which reached the MII stage. N: total number of cultivated oocytes in each group.

Group	MII % (n/N)
CONTROL	27.8 (30/108)*
G 1	49.0 (48/98)*,†
G 2	44.3 (43/97)*,†
G 3	50.5 (49/97)*,†

* Significant differences (*p*>0.05) between control and treated groups.

† no significant differences between groups.

The percentage of survival was also determined for all groups, and the results are presented in Table 2. In the control group, the result was 92.6% (100 oocytes survived out of 108), G1 had a result of 91.8% (90/98); G2 presented a rate of 94.8% (92/97) and the rate of G3 was 95.9% (93/97). There were no significant differences between the groups.

**Table 2:** Survival rates of mouse oocytes. Number of intact oocytes (n) after 24h of IVM. N: total number of cultivated oocytes in each group.

N: total number of cultivated oocytes in each group. Groups	Survival rate % (n/N)
CONTROL	92.6 (100/108)†
G 1	91.8 (90/98)†
G 2	94.8 (92/97†
G 3	95.9 (93/97)†

† no significant differences between groups.

## DISCUSSION

Our results showed that a hyperosmotic shock, induced by short exposure of immature oocytes to vitrification and devitrification solutions, is able to significantly improve *in vitro* maturation up to the MII stage. The prepubescent mice used in this study were not submitted beforehand to ovarian hyperstimulation, since we wanted to simulate the situation in which the patients would not receive any type of hormonal treatment. The fact that IVM results are not influenced by a preparatory ovarian stimulation has been recognized since early trials (Hatırnaz *et al*., 2018; Söderström-Anttila *et al*., 2005), and this suggests that the activation mechanism of oocyte maturation is not solely controlled by endocrine mechanisms.

Another important finding of our study is that the osmotic treatment with commercially available vitrification solutions has no impact on the survival rates of the oocytes during the 24h of *in vitro* maturation. In our protocol, the exposure to the vitrification solution was reduced to a short (30 sec) treatment with the most concentrated vitrification solution (containing 1.4M sucrose). In these conditions, the oocytes are submitted to important osmotic stress, but this did not notably increase lethal cellular injury as one might have expected (Elliott *et al*., 2017). Immature silver fox oocytes were shown to mature equally well, independently whether they were primarily exposed or not to an equilibrium solution before being exposed to the vitrification solution (Cao *et al*., 2017). Similar observations were made with human immature oocytes from IVF patients which matured better after the hyperosmotic shock, induced by vitrification solutions (Molina *et al*., 2016).

Our observations on oocytes *in vitro* maturation from prepubescent mice ovaries behaved similarly to those from adults in other species, probably because they are under the control of similar mechanisms. The most prominent candidate is calcium. Meiosis resumption occurs mainly following an increase in intracellular calcium (Carafoli, 2002). Both cryoprotective substances present in the vitrification medium used in this study have the capacity to enhance calcium exchanges, DMSO acting on the intracellular concentrations, while EG promotes calcium influx from the external medium (Larman *et al*., 2006). The intracellular pH and calcium oscillations induced by the vitrification solution are likely to be tightly associated during oocyte maturation and fertilization. In the oocyte, the pH regulating mechanism seems first at rest and it then becomes activated during maturation and fertilization (FitzHarris & Baltz, 2009). Some pH regulators are sensitive to calcium (or its pathways) because the reactivation of pH regulation corresponds to the beginning of ion oscillations (Jones *et al*., 1995; Marangos *et al*., 2007). Thus, pH homeostasis and regulation are essential partners of calcium during oocyte growth and maturation (FitzHarris & Baltz, 2009).

The process of dehydration-rehydration used in this study is controlled by the selective permeability of the plasma membrane to permeant cryoprotectants (Castro *et al*., 2011) and non-permeant substances able to generate an osmotic gradient (Finan & Guilak, 2010). During devitrification, cryoprotectants are removed, and the cell recovers its volume through the influx of water until osmotic equilibrium is reached (Ambrosini *et al*., 2006; Si *et al*., 2006). Type and concentration of cryoprotectants, exposure time and medium temperature are critical factors that affect the viability of these processes (Liu *et al*., 2012).

Our study highlights a third important aspect associated with the rehydration process. As shown in Table 1, oocytes from G3 had the highest maturation rate compared to the control or to groups 1 and 2. The particular aspect of G3 is that the rehydration, following the hyperosmotic shock, was performed in two steps. It thus appears that the recovery of an iso-osmotic equilibrium with the culture medium is a sensitive process that cannot be solely controlled by time as it involves also thorough and gentle removal of the largest possible portion of the cryoprotectants.

The successful spontaneous maturation of control oocytes (GC) is likely due to the dismantling of the *cumulus oophorus,* and rupturing of the gap-junctions (Vozzi *et al*., 2001), which occur during the collection procedure (Thomas *et al*., 2004). The mechanical recovery of oocytes leads to the recovery of a heterogeneous population of immature oocytes, and the osmotic-shock induced oocyte maturation probably acts on a subpopulation of oocytes that are not activated by the simple dissociation of the cumulus cells.

However, oocyte exposure to cryoprotectants leads to the hardening of the zona pellucida (Larman *et al*., 2006; Matson *et al*., 1997). This is due to the conversion of the zona pellucida glycoprotein (ZP2) into a modified form that is induced by the calcium surge. This phenomenon is normally present after fertilization in order to harden the zona pellucida and prevent polyspermy (Rogers *et al*., 2018). For reproductive purposes, this problem can be circumvented by intracytoplasmic injection (ICSI), which has become a technique of choice for cryopreserved oocytes, since it yields a higher fertilization rate than conventional *in vitro* fertilization (IVF) (Kazem *et al*., 1995).

Regarding toxicity, another negative effect of cryoprotectants (EG and DMSO) is the generation of free radicals (Best, 2015). Antioxidant treatments have been shown to reduce the oxidative damage during the vitrification of immature oocytes in mice (Moawad *et al*., 2014) and pigs (Gupta *et al*., 2010), which suggests that these substances might become routinely used to prevent oxidative damages by cryoprotectants in the future.

Finally, large oscillations in the oocyte maturation responses were observed from one experiment to another (Figure 2). Many factors may be involved in these alterations, such as the status of each animal, environmental alteration, management practices, temperature, feeding, and water intake. The induction of chronic stress in animals is known to trigger a series of hormonal alterations, and cause reproductive problems (Macedo *et al*., 2012; Macfarlane *et al*., 2000). Larger temporal trends during winter and summer are also known to affect maturation rates in bovines (Pavani *et al*., 2017), but most of these effects should have been controlled in our animal facilities.

**Figure 2:** Box and whiskers plot of the percentage of oocyte reaching the metaphase II stage in the 4 groups tested in 11 repeats of the experiments. Control: no treatment, G1, G2, G3: treated groups (see figure 1). Boxes represent p25, p50, and p75; whiskers indicate positions of minimum and maximum values.

## CONCLUSION

In conclusion, the use of commercially available vitrification solutions to induce a hyperosmotic shock did not interfere with the resumption of meiosis in mice oocytes. Further studies are needed to better explain the biological mechanisms involved, to reduce collateral damages caused by the cryoprotectants and to check the ability of such *in vitro* matured oocytes to fertilize.
